# Systematic Analysis of Phosphotyrosine Antibodies Recognizing Single Phosphorylated EPIYA-Motifs in CagA of Western-Type *Helicobacter pylori* Strains

**DOI:** 10.1371/journal.pone.0096488

**Published:** 2014-05-06

**Authors:** Judith Lind, Steffen Backert, Klaus Pfleiderer, Douglas E. Berg, Yoshio Yamaoka, Heinrich Sticht, Nicole Tegtmeyer

**Affiliations:** 1 Friedrich Alexander University Erlangen-Nuremberg, Department of Biology, Division of Microbiology, Erlangen, Germany; 2 Division of Infectious Disease, Department of Medicine, University of California San Diego, La Jolla, California, United States of America; 3 Oita University Faculty of Medicine, Department Environmental and Preventive Medicine, Yufu, Japan; 4 Friedrich Alexander University Erlangen-Nuremberg, Bioinformatics, Institute for Biochemistry, Erlangen, Germany; Institut Pasteur Paris, France

## Abstract

The clinical outcome of *Helicobacter pylori* infections is determined by multiple host-pathogen interactions that may develop to chronic gastritis, and sometimes peptic ulcers or gastric cancer. Highly virulent strains encode a type IV secretion system (T4SS) that delivers the effector protein CagA into gastric epithelial cells. Translocated CagA undergoes tyrosine phosphorylation at EPIYA-sequence motifs, called A, B and C in Western-type strains, by members of the oncogenic Src and Abl host kinases. Phosphorylated EPIYA-motifs mediate interactions of CagA with host signaling factors – in particular various SH2-domain containing human proteins – thereby hijacking multiple downstream signaling cascades. Observations of tyrosine-phosphorylated CagA are mainly based on the use of commercial phosphotyrosine antibodies, which originally were selected to detect phosphotyrosines in mammalian proteins. Systematic studies of phosphorylated EPIYA-motif detection by the different antibodies would be very useful, but are not yet available. To address this issue, we synthesized phospho- and non-phosphopeptides representing each predominant Western CagA EPIYA-motif, and determined the recognition patterns of seven different phosphotyrosine antibodies in Western blots, and also performed infection studies with diverse representative Western *H. pylori* strains. Our results show that a total of 9–11 amino acids containing the phosphorylated EPIYA-motifs are necessary and sufficient for specific detection by these antibodies, but revealed great variability in sequence recognition. Three of the antibodies recognized phosphorylated EPIYA-motifs A, B and C similarly well; whereas preferential binding to phosphorylated motif A and motifs A and C was found with two and one antibodies, respectively, and the seventh anti-phosphotyrosine antibody did not recognize any phosphorylated EPIYA-motif. Controls showed that none of the antibodies recognized the corresponding non-phospho CagA peptides, and that all of them recognized phosphotyrosines in mammalian proteins. These data are valuable in judicious application of commercial anti-phosphotyrosine antibodies and in characterization of CagA phosphorylation during infection and disease development.

## Introduction

Posttranslational modification of proteins by kinases is important in many cell signaling processes. Although phosphorylation of some serine, threonine and histidine residues occurs both in prokaryotes and eukaryotes, tyrosine phosphorylation is believed generally to be mostly restricted to higher organisms, where it plays important roles in signal transduction and developmental regulation [1]. In fact, typical tyrosine kinase genes have been reported in only very few sequenced bacterial genomes [2], [3]. However, there are numerous reports of effector proteins from pathogenic bacteria that undergo tyrosine phosphorylation after translocation into eukaryotic host cells, which is a remarkable example of convergent evolution, not just descent from a common ancestor [2], [4]–[6]. In various cases, effector protein phosphotyrosines together with some flanking residues act as recognition motifs for eukaryotic signaling factors. They recruit in particular cellular binding partners that contain SH2 (Src homology 2) domains, but not PTB (phosphotyrosine binding) domains, and thereby target and subvert eukaryotic signal transduction pathways in ways that benefit the pathogen [2], [4]. This virulence strategy is well-established for six different bacterial pathogens: enteropathogenic *Escherichia coli* (EPEC), *Helicobacter pylori, Chlamydia trachomatis*, *Bartonella henselae*, *Anaplasma phagocytophilum* and *Ehrlichia chaffeensis* [7]–[13].

The virulence factor CagA of the gastric pathogen *H. pylori* provides a prime example of such tyrosine phosphorylatable effector proteins [8], [14]–[18]. CagA is delivered to host cells via a type IV secretion system (T4SS), a complex syringe-like pilus device whose synthesis is encoded in the *cag* pathogenicity island and induced on contact with target cells [19]–[22]. A hallmark of cultured AGS gastric epithelial cells infected by CagA-producing *H. pylori* strains is the development of the so-called “hummingbird” or “elongation” cell phenotype [8], [23], [24]. This *in vitro* phenotype is likely to reflect several *in vivo* signaling processes that control immune responses, wound healing, metastasis and invasive growth of cancer cells [25], [26]. CagA interacts with more than 20 host cell proteins, variously in phosphorylation-dependent and phosphorylation-independent manners [5]. Sequence analysis and site-directed mutagenesis identified a series of EPIYA (Glu-Pro-Ile-Tyr-Ala) motifs near the CagA carboxy-terminus as phosphorylation sites and showed that phospho-CagA is essential for AGS cell elongation [23], [24], [27]–[30]. Four specific EPIYA-motifs termed A, B, C and D have been identified based primarily on relative positions in CagA and adjoining amino acid sequences despite some diversity in flanking sequences and even in EPIYA-motifs themselves [5], [6], [31]-[33]. Whereas EPIYA-A and EPIYA-B motifs are found in all CagA proteins, EPIYA-C is mainly found in strains of African and Indo-European ancestry, whereas CagA from most East-Asian strains contain the more potent EPIYA-D motif in place of EPIYA-C. Although most CagA proteins contain only three EPIYA-motifs, some strains have additional EPIYA-copies [5], [6], due to recombination between repetitions in flanking DNA sequences [31], [34]–[44]. Two-dimensional gel electrophoresis (2-DE) of phospho-CagA proteins from infections of AGS or MKN-28 cells by Western *H. pylori* strains with 3-4 EPIYA-motifs has shown that only one or two tyrosines (but not three) can be phosphorylated per CagA molecule [45], [46].

The host tyrosine kinases active on these CagA EPIYA-motifs were identified as members of the Src [24], [47] and Abl [48], [49] families. We found that c-Src only phosphorylated EPIYA-C or EPIYA-D, while c-Abl phosphorylated EPIYA-A, EPIYA-B, EPIYA-C, and EPIYA-D. Further analysis revealed that none of the phosphorylated EPIYA-motifs alone was sufficient for inducing AGS cell elongation [46]. Site-directed mutagenesis has shown that the preferred combination of phosphorylated EPIYA-motifs in Western strains was EPIYA-A and EPIYA-C, either across two CagA molecules or simultaneously on one [46]. These studies thus identified a tightly regulated hierarchic phosphorylation model for CagA starting at EPIYA-C/D, followed by phosphorylation at EPIYA-A or EPIYA-B. However, the observation that CagA can undergo tyrosine phosphorylation in host cells is mainly based on the use of commercial α-phosphotyrosine antibodies in Western blots [8], [14]–[17]. These antibodies had been selected years ago to specifically detect a broad range of phosphorylated tyrosine residues in mammalian proteins. Three of these phosphotyrosine-specific antibodies have been shown to exhibit a similar phosphotyrosine-binding preference in mammalian proteins, preferably with a proline residue at position +3 and a leucine at position -1 [50]. However, proline and leucine residues are not present at this position in the corresponding phosphorylation sites of CagA [2], [5], [6]. In addition, systematic studies on the specific recognition patterns of phosphotyrosine motifs in the delivered bacterial effectors such as CagA by a large number of different antibodies are not yet available. Therefore, we addressed this important question and synthesized phospho- and non-phospho peptides of each CagA EPIYA-motif from Western strains to investigate the recognition specificity by seven commercially available phosphotyrosine antibodies. We also performed infection studies with *H. pylori* to investigate the recognition patterns of phosphorylated CagA upon delivery into host target cells.

## Materials and Methods

### Bacterial strains and culture conditions

All wild-type *H. pylori* strains were typical type-I isolates expressing CagA. The generation of an isogenic Δ*cagA* mutant has been described [17]. *H. pylori* was grown in thin layers on horse serum GC agar plates supplemented with vancomycin (10 µg/mL), nystatin (1 µg/mL), and trimethoprim (5 µg/mL) as described previously [51], [52]. All antibiotics were obtained from Sigma-Aldrich (St. Louis, MO, USA). Bacteria were grown at 37°C for 2 days in an anaerobic jar containing a Campygen gas mix of 5% O_2_, 10% CO_2_, and 85% N_2_ (Oxoid, Wesel, Germany) [53], [54].

### Synthesis of phospho- and non-phospho CagA peptides

The C-STEPIYAKVNK (EPIYA-A), C-STEPI(pY)AKVNK (phospho-EPIYA-A), C-PEEPIYTQVAK (EPIYA-B), C-PEEPI(pY)TQVAK (phospho-EPIYA-B), C-SPEPIYATIDD (EPIYA-C) and C-SPEPI(pY)ATIDD (phospho-EPIYA-C) sequences were synthesized by Jerini AG (Berlin, Germany) and the C-TEPI(pY)AKVN, C-EPI(pY)AKV and C-PI(pY)AK peptides by Biosyntan GmbH (Berlin, Germany). These 11-mer peptides were chosen to compare the three EPIYA-motifs because α-phosphotyrosine antibodies typically recognize short phosphopeptides [35], [50], [55], [56]. Commonly, 11-mer peptides are also used for immunizations to generate phospho-specific antibodies, which then recognize the corresponding phosphopeptides bound to affinity columns and in ELISA (Biogenes, Berlin, Germany). All above EPIYA peptides were purified by HPLC, and full-length synthesis as well as purity of each peptide was confirmed by mass spectrometry by Jerini AG and Biosyntan AG. The peptides were resolved at a concentration of 1 mg/mL in DMSO and stored at −20°C.

### Cloning and purification of recombinant CagA

A *cagA* gene fragment of 891 bp (corresponding to amino acid positions 890-1,186 in the C-terminus of CagA from *H. pylori* strain 26695) including the EPIYA-motifs A, B and C was synthesized by Geneart (Regensburg, Germany). This *cagA* fragment was then subcloned into the pGEX-2T vector using the restriction enzymes *Bam*HI and *Eco*RI. The resultant construct was transformed into the *E. coli* strain BL21. Protein expression was carried out in 800 mL of pre-warmed LB medium, which were inoculated with 8 mL of an overnight culture. When cells reached an OD_600 nm_ of 0.4, protein expression was induced with 1 mM IPTG. After 4 hours, the cells were harvested and the pellet was stored at −20°C. Prior to cell disruption by sonication, the pellet was suspended in 30 mL PBS (phosphate buffered saline) supplemented with 1 mM DTT. To remove cell debris, the sample was centrifuged at 25,000 rpm for 50 min. Subsequently, the supernatant was loaded onto a 1 mL GSTrap HP column (GE Healthcare, Munich, Germany) and bound target protein was eluted with 50 mM Tris-HCl pH 8.0 containing 10 mM reduced Glutathione and 1 mM DTT. Fractions were analyzed by SDS-PAGE and Western blotting. Selected CagA-positive fractions were pooled and further purified using HiLoad 16/60 Superdex 75 (GE Healthcare) equilibrated with 20 mM Tris-HCl pH 8.0, 150 mM NaCl and 1 mM DTT. Peak fractions were analyzed by SDS-PAGE and Western blot. Fractions containing the purified CagA fragment showed no detectable impurities by other proteins.

### *In vitro* phosphorylation of CagA with recombinant c-Abl kinase

10^10^ cells of *H. pylori* strain 26695 expressing wild-type CagA (or isogenic Δ*cagA* mutant as control) were harvested in 1 mL of kinase buffer as described previously [47]. A total of two units of recombinant human c-Abl tyrosine kinase (NEB GmbH, Frankfurt/M., Germany) and 1 µmol/L of ATP were mixed with 30 µL *H. pylori* lysate or 10 µL recombinant CagA and incubated for 30 min at 30°C as described previously [49]. The reactions were terminated by a 5 min denaturing step at 95°C.

### Dotblot analysis

Twenty µg of each CagA peptide or 30 µl of the *in vitro* kinase reaction products described above were mixed in 1 mL of blotting buffer (192 mM Glycin; 20 mM Tris-HCl, pH 8,4; 0.1% SDS; 20% Methanol). These peptide samples were spotted onto Immobilon-P membrane (Merck Millipore, Darmstadt, Germany) using the BioDot SF apparatus (Bio-Rad, Munich, Germany). The resulting Dotblots were dried and subjected to antibody detection as described below for Western blots.

### Eukaryotic cell culture and elongation phenotype quantitation assays

Human adherent gastric adenocarcinoma epithelial cells (AGS, ATCC CRL-1730) were grown in 6-well plates containing RPMI 1640 medium (Invitrogen) supplemented with 25 mM HEPES buffer and 10% heat-inactivated FBS (Biochrom, Berlin, Germany) for 2 days to approximately 70% confluence [57], [58]. Cells were serum-deprived overnight and infected with *H. pylori* at a MOI of 50 for 6 hours. After infection, the cells were harvested in ice-cold PBS containing 1 mmol/L Na_3_VO_4_ (Sigma-Aldrich). Elongated AGS cells in each experiment were quantitated in 10 different 0.25-mm^2^ fields using an Olympus IX50 phase contrast microscope. All experiments were performed in triplicate and subjected to statistical analysis as described below.

### SDS-PAGE and immunoblot analysis

AGS cell pellets with attached bacteria were mixed with equal amounts of 2 x SDS-PAGE buffer and boiled for 5 minutes. Proteins were separated by SDS-PAGE on 6% polyacrylamide gels and blotted onto PVDF membranes (Immobilon-P, Merck Millipore). Membranes were blocked in TBST with 3% BSA or 5% skim milk for 1 hour at room temperature. Membranes were incubated with the seven α-phosphotyrosine antibodies (Table 1) or mouse monoclonal α-CagA antibody (Austral Biologicals, San Ramon, CA, USA) according to the instructions of the manufacturer. Phosphorylated and non-phosphorylated CagA proteins were detected using horseradish peroxidase–conjugated anti-mouse or anti-rabbit polyvalent sheep immunoglobulin secondary antibodies in the ECL Plus chemoluminescence Western blot system of GE Healthcare [59]–[62].

**Table 1:** Characteristics of commercial α-phosphotyrosine antibodies used in this study.

Antibody Name	Short name^a^	Origin/isotype	Used antigen(s)	Given information on antibody specificity	Dilution used	Order number	Company
p-Tyr (PY99)	α-PY-99	mouse-mAB-IgG2b	np	no cross reactivity with Phospho-Ser or Phospho-Thr	1∶1,000	sc-7020	Santa Cruz Biotechnology
Anti-phosphotyrosine (clone PY20)	α-PY-20 (BD)	mouse-mAB-IgG2b	np	np	1∶500	61000	BD Biosciences
p-Tyr (PY20)	α-PY-20 (SC)	mouse-mAB-IgG2b	np	np	1∶1,000	sc-508	Santa Cruz Biotechnology
Phospho-Tyrosine Mouse mAB (P-Tyr-100)	α-PY-100	mouse-mAB-IgG1	mix of phospho-tyrosine peptides (np)	no cross reactivity with Phospho-Ser or Phospho-Thr	1∶1,000	9411	Cell Signaling
Mouse anti-phospho-tyrosine (clone PY69)	α-PY-69	mouse-mAB-IgG2a	np	np	1∶1,000	610430	BD Biosciences
Phospho-Tyrosine Mouse mAB (P-Tyr-102)	α-PY-102	mouse-mAB-IgG2	mix of phospho-tyrosine peptides (np)	no cross reactivity with Phospho-Ser or Phospho-Thr	1∶1,000	9416	Cell Signaling
p-Tyr (PY350)	α-PY-350	rabbit-pAB-IgG	np	no cross reactivity with Phospho-Ser or Phospho-Thr	1∶500	sc-18182	Santa Cruz Biotechnology

Abbreviations: IgG (immunoglobulin G); mAB (monoclonal antibody); np (information not provided by the company); pAB (polyclonal antibody); p-Tyr, PY (phosphotyrosine); Ser (serine); Thr (threonine); Tyr (tyrosine).

a short name used in this study.

### Quantification of Dotblot and Western blot signals

Spot or band intensities on blots probed with the different α-phosphotyrosine antibodies were quantitated with the Lumi-Imager F1 (Roche Diagnostics, Mannheim, Germany). Densitometric measurement of signal intensities revealed the percentage of phosphorylation per sample [63]. The strongest spot on Dotblots was set at 100% as indicated in the corresponding Figures.

### Statistical analysis

All data were evaluated using Student t-test with SigmaStat statistical software (version 2.0). All error bars shown in figures and those quoted following the +/− signs represent standard deviations.

## Results

### Strong recognition of 9-mer and 11-mer CagA phosphopeptides by α-phosphotyrosine antibodies

The majority of CagA proteins in Western type clinical isolates contain three EPIYA-motifs, such as that of the first fully sequenced *H. pylori* strain 26695 (Figure 1A). Commercial phosphotyrosine antibodies typically recognize short mammalian phosphopeptides; in some cases even five amino acids were previously shown to be sufficient for recognition [35], [50], [55], [56]. To systematically analyze the recognition capabilities of phosphorylated CagA EPIYA-motifs by α-phosphotyrosine antibodies we first synthesized a series of peptides derived from the EPIYA-A motif exhibiting the phosphotyrosine residue in the middle +/− five, four, three or two flanking amino acids, including the STEPIYAKVNK (11-mer), TEPIYAKVN (9-mer), EPIYAKV (7-mer) and PIYAK (5-mer) sequences as indicated (Figure 1B, top). Twenty µg of each EPIYA-peptide was immobilized per spot on PVDF membranes using the Dotblot method followed by probing with the α-phosphotyrosine antibodies α-PY99 and α-PY20 (BD). The results show that both antibodies recognized 11-mers and 9-mers with similar strong intensity, while recognition of 7-mers and 5-mers was significantly reduced (Figures 1B). An 11-mer of the corresponding non-phospho-EPIYA peptide did not produce signals in a parallel control experiment (Figure 1B). In further tests, the efficient Dotblot approach detected full-length CagA in bacterial lysates or recombinant C-terminal CagA when phosphorylated by c-Abl in *in vitro* kinase reactions (Figure 1C). This experiment also confirmed that the α-phosphotyrosine antibodies do not cross-react with non-phospho CagA proteins in control reactions without c-Abl kinase (Figure 1C and data not shown), as expected.

**Figure 1:** Short EPIYA-phosphopeptides of *H. pylori* CagA are sufficient for detection by α-phosphotyrosine antibodies. (**A**) Typical Western CagA proteins of *H. pylori* such as that of strain 26695 [76] contain the EPIYA-A, EPIYA-B, and EPIYA-C segments as indicated. These motifs represent tyrosine phosphorylation sites, which can be phosphorylated by c-Abl and c-Src host kinases. (**B**) The indicated phospho- and non-phospho peptides of the EPIYA-A motif were synthesized and immobilized on PVDF membranes using a Dotblot apparatus. All Dotblots were probed with the indicated commercial phosphotyrosine antibodies and exposed as described in the Material & Methods section. Quantified spot intensities of the Dotblots from three independent experiments are shown to the right. Signal intensities were measured densitometrically with the Lumi-Imager F1 and revealed the percentage of phosphorylation signal per sample. The strongest spot on every Dotblot was set at 100% for each of the different α-phosphotyrosine antibodies as indicated. The results show that 11-mer and 9-mer phosphopeptides are sufficient for strong recognition by the antibodies. (**C**) Control Dotblot analyses used products of *in vitro* kinase reactions of c-Abl with either bacterial lysates (from *H. pylori* wild-type strain 26695 and isogenic Δ*cagA* mutant) or a purified recombinant CagA C-terminal fragment. Phosphorylated CagA proteins can be also detected by this Dotblot method using seven phosphotyrosine antibodies (Table 1), while the non-phosphorylated CagA forms cannot.

### Recognition of phosphopeptides from EPIYA-A, -B and -C by α-phosphotyrosine antibodies

After validating the Dotblot approach using phospho-CagA peptides functions, we synthesized 11-mer phospho- and non-phosphopeptides of EPIYA-B (PEEPIYTQVAK) and EPIYA-C (SPEPIYATIDD) motifs as indicated (Figure 2A, top) and probed them with a set of seven different commercially available α-phosphotyrosine antibodies (Table 1). The results confirmed that these antibodies do not cross-react with the corresponding non-phospho CagA peptides (Figure 2A), and showed, interestingly, that all antibodies except α-PY350 predominantly recognized the EPIYA-A phosphopeptide, which did not recognize any of the CagA-derived phosphopeptides. Some remarkable differences, however, were seen in the abilities of the antibodies to react with the EPIYA-B and EPIYA-C phosphopeptides. In particular, three antibodies (α-PY99, α-PY20-BD, α-PY20-SC) recognized all three phosphorylated EPIYA-A, EPIYA-B and EPIYA-C peptides with similar strong signals, while two others (α-PY100, α-PY69) recognized the phosphorylated EPIYA-A peptide preferentially, and phospho-EPIYA-B and phospho-EPIYA-C more weakly (Figure 2A). A sixth antibody (α-PY102) recognized phosphorylated EPIYA-A strongly and EPIYA-C very weakly, while the seventh antibody, α-PY350, did not recognize any phosphorylated EPIYA-peptide, as noted above (Figure 2A). This inability to detect signals with the α-PY350 antibody was unaffected by binding five-fold more peptide (0.1 mg) to membranes or use of twice as much antibody (data not shown), even though we confirmed that our batch of α-PY350 effectively recognizes phosphorylated host proteins, as discussed below. The quantification of Dotblot data from three independent experiments is presented in Figure 2B. Taken together, the results revealed enormous variability in the capability of seven α-phosphotyrosine antibodies to recognize phosphorylated EPIYA-motifs A, B and/or C.

**Figure 2:** Variable recognition of synthetic 11-mer CagA phospho-peptides by seven commercial α-phosphotyrosine antibodies. (**A**) Dotblot analysis of the indicated phospho- and non-phospho peptides derived from single EPIYA-motifs A, B and C. All Dotblots were probed with the indicated commercial phosphotyrosine antibodies and exposed as described in the Material & Methods section. (**B**) Quantification of spot intensities on Dotblots. Signal intensities were measured densitometrically with the Lumi-Imager F1 and revealed the percentage of phosphorylation signal per sample. The strongest spot on every Dotblot was set at 100% for each of the different α-phosphotyrosine antibodies as indicated. Quantitation results are shown for three independent experiments.

### Recognition of phosphorylated CagA protein during infection of AGS cells

Next, we aimed to investigate recognition patterns of phosphorylated CagA proteins during infection. For this purpose, we selected eight representative *H. pylori* strains from different continents, including Africa, Europe, Asia, North America and South America (Table 2). Sequence alignment of CagA carboxy-terminal regions establishes that all three EPIYA-motifs A, B and C are present, although with some heterogeneity in flanking amino acid sequences (Figure 3). AGS cells were infected for 6 hours with these *H. pylori* strains and the elongation phenotype of infected cells was monitored over time, to indicate successful CagA delivery and phosphorylation [64]–[66]. About 60−70% of AGS cells exhibited the elongation phenotype after infection with each *H. pylori* strain, suggesting that high amounts of phospho-CagA are produced (Figure 4). Next, protein lysates were prepared from infected AGS cells and analyzed with the different antibodies. First, the samples were probed with a monoclonal α-CagA antibody recognizing both non-phosphorylated and phosphorylated forms of CagA, to ensure that similar amounts of CagA protein were loaded in each lane (Figure 5, top). The various CagA variants exhibit different band sizes between 130−150 kDa as expected from the different strains (Table 2). The samples were then probed with the seven α-phosphotyrosine antibodies. The results confirmed that all antibodies recognized host cell proteins (Figure 5, asterisks), whereas phospho-CagA was recognized by only some of the antibodies (Figure 5, arrows). The quantification data for phospho-CagA from three independent experiments are presented in Table 3. Two antibodies (α-PY99 and α-PY20-BD) produced strong phospho-CagA bands from all eight strains with little background in the 125−150 kDa region (Figure 5). This indicates that sufficient detectable phospho-CagA was generated during infection and confirmed the elongation phenotype data for each strain noted above. Interestingly, phospho-CagA from two strains (26695 and Sat464) was strongly recognized by six of the seven α-phosphotyrosine antibodies. Antibodies α-PY20-SC, α-PY100 and α-PY102, which recognized all three phospho-EPIYAs in the above Dotblots gave mixed results. Although these three antibodies produced strong bands with phospho-CagA from *H. pylori* strains 26695 and Sat464, they produced only weak signals with phospho-CagA from strains P310, Lit75, B8, 2002-370 and Oki61 (Figure 5). In addition, it should be noted that the phospho-CagA patterns among these three antibodies were not identical. For example, phospho-CagA from strain Gam94/24 was strongly recognized by α-PY20-SC, but only weakly by α-PY100 and not by α-PY102. The seventh antibody, α-PY350, did not recognize phosphorylated CagA from any *H. pylori* strain tested, in agreement with results obtained using EPIYA phosphopeptides, although it did recognize major 125, 150 and 170 kDa host phosphoproteins (Figure 5, bottom). Antibody α-PY69 also appears to be not very useful for studying CagA phosphorylation in AGS cells because of the presence of a cross-reacting host phosphoprotein at about 140 kDa, which is in the size range of various phospho-CagA bands (Figure 5).

**Figure 3:** Sequence comparison of the EPIYA-motifs in CagA proteins from different clinical *H. pylori* strains used in the study. Western CagA proteins of *Helicobacter pylori* vary in the carboxy-terminal phosphorylation sites EPIYA-A, EPIYA-B, and EPIYA-C depending on their geographical origin. These EPIYA-repeats serve as tyrosine phosphorylation sites of CagA and can be targeted by c-Abl and c-Src kinases [24], [30], . Multiple EPIYA-segments A, B and C are shaded with yellow and variations in the flanking regions were found among clinical *H. pylori* isolates from different continents as indicated. One striking feature of EPIYA-B (and in some strains in EPIYA-A) is the presence of a negatively charged glutamate residue in the -4 position (shaded with green), which is highly conserved in EPIYA-B among the different *H. pylori* strains and may affect the binding capabilities of phosphotyrosine antibodies as discussed in the text. The CagA protein sequences were obtained from databases (Table 2) and sequence alignment was done using the ClustalW2 program (http://www.ebi.ac.uk/Tools/msa/clustalw2/).

**Figure 4:** AGS cell elongation induced during infection with different clinical *H. pylori* strains. AGS cells were infected for 6-expressing *H. pylori* strains as indicated. (**A**) The number of elongated cells in each experiment was quantitated in triplicate in 10 different 0.25-mm^2^ fields [77]–[79]. (**B**) Representative phase contrast micrographs of AGS cells infected with the different strains as indicated.

**Figure 5:** Role of EPIYA motifs in CagA phosphorylation during *H. pylori* infection was investigated with seven different α-phosphotyrosine antibodies. AGS cells were infected for 6-expressing *H. pylori* strains as indicated. The samples in Figure 4 were harvested after photographing. Phosphorylation of CagA was examined using the indicated α–phosphotyrosine antibodies. Loading of equal amounts of CagA from each sample was confirmed by probing with a monoclonal α-CagA antibody. A larger section of the ∼120−180 kDa range is shown and contains the phospho-CagA bands of different sizes (arrows) as well as a set of tyrosine-phosphorylated host cell proteins (red asterisks). The blue asterisk indicates a putative N-terminal fragment of CagA which sometimes appears on SDS-PAGE gels [23].

**Table 2:** Characteristics of *H. pylori* strains and encoded CagA proteins used in this study.

H. pylori strain	Origin	Pathology	CagA EPIYA type	Accession Number	Reference
26695	UK	Gastritis	ABC	NP_207343.1	[76]
P310	Germany	Gastric cancer	ABC	AAY18598	[80]
Lit75	Lithuania	Non-atrophic gastritis	ABC	YP_005772684	D. Kersulyte and D. Berg (unpublished)
B8	USA	Peptic ulcer	ABC	FN598874.1	[81]
2002−370	Mexico	Non-atrophic gastritis	ABC	JN390443	[46]
Sat464	Peruvian Amazon	Not evaluated directly [Non-atrophic gastritis assumed]	ABC	YP_005768457	D. Kersulyte and D. Berg (unpublished)
Gam94/24	Gambia	Not evaluated directly [Non-atrophic gastritis assumed]	ABC	YP_005780282	D. Kersulyte and D. Berg (unpublished)
Oki61	Japan	Duodenal ulcer	ABC	AB725848	[82]

**Table 3:** Recognition of EPIYA-phosphopeptides and phosphorylated CagA proteins by commercial α-phosphotyrosine antibodies.

Phospho-antibody name	Recognition of phosphopeptides			Phosphorylation signal intensity of translocated CagA by *H. pylori* strains							
	EPIYA-A	EPIYA-B	EPIYA-C	26695	P310	Lit75	B8	2002-370	Gam94/24	Sat464	Oki61
α-PY-99	+++	+++	+++	+++	+++	+++	+++	+++	+++	+++	+++
α-PY-20 (BD)	+++	++	++	+++	+++	+++	+++	+++	+++	+++	+++
α-PY-20 (SC)	+++	++	++	++	++	++	++	++	+++	+++	++
α-PY-100	+++	+	++	++	++	++	++	+	++	+++	++
α-PY-69	+++	+	+	+++	+/−	+/−	+/−	+/−	++	+++	++
α-PY-102	+++	−	+	+++	++	++	++	−	−	++	++
α-PY-350	−	−	−	−	−	−	−	−	−	−	−

Abbreviations used: PY (phosphotyrosine); EPIYA motif (*glutamic acid*-proline-isoleucine-tyrosine-alanine phosphorylation motif in CagA),

Antibody recognition: +++ (strong signal); ++ (moderate signal); + (weak signal); − (no signal).

### Phospho-EPIYA recognition patterns are influenced both by length and amino acid sequence

The binding specificities of the α-PY20 and α-PY100 antibodies have been experimentally characterized using microarrays of phosphopeptide libraries derived from mammalian proteins [50]. This knowledge allowed to investigate the sequence features responsible for differences in binding affinity observed for the EPIYA-B phosphopeptide in more detail. This peptide is recognized by α-PY100 with lower affinity, whereas the other phosphopeptides (EPIYA-A and EPIYA-C) are recognized by α-PY20 and α-PY100 with similar affinity (Figure 1, Table 3). One striking feature of phospho-EPIYA-B is the presence of a negatively charged glutamate residue in the -4 position, which is highly conserved in CagA among different *H. pylori* strains (Figure 3, shaded with green). The peptide array data from Tinti and co-workers [50] indicates that the presence of a glutamate at this position negatively affects α-PY100 binding, but not α-PY20 binding. Thus, the differences in α-PY20 and α-PY100 binding of phospho-EPIYA-B in our experiments are in line with data from mammalian phosphoproteins and can most likely be attributed to this sequence position. In addition, phosphorylated CagA from different *H. pylori* strains during infection is generally detected better by α-PY20 than by α-PY100 (Figure 5 and Table 3). These differences in α-PY100 binding most likely result from strain-specific sequence variations in the vicinity of the EPIYA-A motif, which is generally less well-conserved than in the vicinity of the EPIYA-motifs B and C (Figure 3). Phospho-CagA produced by the *H. pylori* strains P310 and Gam94/24 is bound by α-PY100 with relatively low affinity (Figure 5), which can be attributed at least in part to a glutamate at the -4 position of the EPIYA-A motif (Figure 3, shaded with green). Further inspection of the overall data in Table 3 suggests that additional features also affect α-PY100 binding specificity, as evidenced by the low affinity of phospho-CagA from *H. pylori* strains B8 and 2002-370 produced during infection. These features are likely determined by residues flanking the EPIYA core motif, as suggested by the significantly weaker binding of the 5-mer and 7-mer peptides described above.

## Discussion

The CagA protein and its EPIYA-motifs are known for long time as important virulence markers of *H. pylori* [5], [6], [18], [23], [24], [27]–[34], [67], [68]. These EPIYA-repeat motifs were originally described in 1993 by the group of Antonello Covacci [69]. Even before these sequences were identified to be the sites of CagA tyrosine phosphorylation [23], certain variations within the EPIYA-region at the sequence level have been reported and associated with gastric disease [70], [71]. After the discovery of CagA tyrosine phosphorylation about 15 years ago [18], intensive efforts were undertaken to identify the involved host cell kinases [5]. Mammals encode about 90 protein tyrosine kinases [72], which phosphorylate their mammalian substrates with specificity depending on amino acid sequences next to the targeted tyrosine residue [73]. The EPIYA-motifs in CagA commonly have isoleucine at the –1 position and the small amino acid alanine at the +1 position, which is similar to the phosphorylation consensus motif EEIYG/E of the host kinase c-Src [47]. Indeed, several lines of evidence have then demonstrated that c-Src and also c-Abl family kinases mediate CagA phosphorylation *in vitro* and *in vivo* [24], [46]–[49], [74]. However, progress in this research field has been hampered by a lack of standardized commercial EPIYA-specific phospho-antibodies and lack of knowledge about which phospho-EPIYAs are recognized by the set of available α-phosphotyrosine antibodies (Table 1). Systematic examination of which phosphotyrosine residues in the three different EPIYA-motifs are recognized by these various antibodies has not yet been reported. Thus, despite the years of research, detailed, clear-cut conclusions about CagA phosphorylation patterns in clinical strains have not been possible. Here, we investigated for the first time the recognition specificity of seven commercially available α-phosphotyrosine antibodies with regard to CagA EPIYA-motifs A, B and C in Western *H. pylori* strains. We found that these antibodies exhibit a remarkable variety in recognition of the various phosphorylated EPIYA-motifs. These results shed light on the usefulness of these antibodies in research and provide valuable new insights for future studies on CagA phosphorylation sites and downstream signaling.

It is well known that the α-phosphotyrosine antibodies were originally developed for mammalian proteins and typically recognize short amino acid stretches containing the phosphorylated tyrosine residue, including synthetic phospho-peptides [35], [50], [55], [56]. We therefore proposed that phospho-peptides derived from the CagA EPIYA-motifs would be useful for studying the recognition capabilities by seven commercial antibodies. Using this strategy we found that 9-mers and 11-mers of EPIYA-phosphopeptides are necessary and sufficient for strong antibody recognition. In addition, three α-phosphotyrosine antibodies (α-PY99, α-PY20-BD and α-PY20-SC) recognized all three 11-mer phospho-EPIYA peptides (A, B and C) with similar and very strong affinity, confirming that this approach works for peptides derived from bacterial effector proteins in addition to mammalian peptides. Overall, this observation nicely correlated with the pronounced recognition of phospho-CagA in cell lysates produced after infection with eight different *H. pylori* strains (Table 3). Another antibody (α-PY100) reacted preferentially with phospho-EPIYA peptides A and C, and also produced acceptable phospho-CagA patterns by Western blotting of extracts from infected cells. In addition, antibody α-PY102 strongly recognized phospho-EPIYA peptide A and very weakly phospho-EPIYA peptide C, but reacted only with six of eight phospho-CagAs in infected cells. Although α-PY69 also recognized phospho-EPIYA-A preferentially (with weak signals for B and C), it also strongly reacted with host cell proteins in the 125–140 kDa range and is therefore not useful for studying CagA phosphorylation during infection. Importantly, the antibodies α-PY99, α-PY20-BD, α-PY20-SC, α-PY100 and α-PY102 did not react with AGS host cell proteins in the 130–150 kDa range, another important criterion that makes them useful for *H. pylori* studies. These results allow us to recommend the use of up to five α-phosphotyrosine antibodies for studies of infection by *H. pylori* (α-PY99, α-PY20-BD and α-PY20-SC, and if needed, also α-PY100 and α-PY69) based on their ability to recognise a broad spectrum of different phospho-CagAs, and thereby to clarify what EPIYAs are phosphorylated.

Most knowledge about phosphotyrosine-based protein-protein interactions is derived from use of α-phosphotyrosine antibodies to investigate mammalian signaling factors [1]. Recent studies have applied the microarray technology to characterize the substrate specificity of widely used α-phosphotyrosine antibodies (including α-PY100 and α-PY20) in human phosphopeptides [50]. The conclusions that were drawn from this analysis are: (i) the antibodies exhibit a similar phosphotyrosine binding specificity whilst at the same time showing specific binding preference depending on some flanking amino acids; and (ii) the similar phosphotyrosine binding specificity is rather broad although proline residues are preferred at position +3 and leucine at position –1 [50]. In addition, the investigations by Tinti and co-workers indicated that the presence of a negatively charged residue such as glutamate at the –4 position specifically affects interaction with α-PY100, but not with α-PY20 [50]. Interestingly, EPIYA-B has a glutamate residue at the –4 position (and sometimes at EPIYA-A), which is highly conserved in CagA among the different *H. pylori* strains (Figure 3). However, inspection of our overall data in Table 3 suggests that additional features also affect α-PY100 binding specificity, as evidenced by the low affinity to phospho-CagA from strains B8 and 2002-370. Both *H. pylori* strains differ at several sequence positions in the vicinity of EPIYA-motif A rendering it difficult to clearly correlate antibody affinity with a single sequence position. This also suggests the existence of other structural features, like secondary structure of the motif and its vicinity, which may additionally affect α-phosphotyrosine antibody binding specificity.

How could one apply this knowledge of binding preferences of α-phosphotyrosine antibodies for certain EPIYA-motifs? The use of α-phosphotyrosine antibodies by probing one-dimensional SDS-PAGE blots of lysates from *H. pylori* infected cells provides a useful first picture of CagA phosphorylation events [75]. However, this picture is not completely useful because increased phospho-CagA signal intensities that can arise over time could result either from increased amounts of translocated CagA molecules undergoing phosphorylation at a specific site, from increased phosphorylation of multiple sites per CagA molecule, or both – possibilities that cannot be distinguished on 1-DE gels. Using 2-DE gel separation of different CagA protein spots, we have recently shown that CagA can be simultaneously phosphorylated either on one or two EPIYAs per molecule [46]. This suggests the appearance of multiple differentially phosphorylated CagA protein species in host cells, each with different functions, and thus could explain how CagA achieves signaling to many different host binding partners [46]. To investigate this hypothesis further and to obtain better tools for clinical applications, it will be desirable in the near future to generate phospho-specific α-CagA antibodies for each EPIYA-motif. In this context, the α-PY69 and α-PY102 antibodies may already be useful because they predominantly detect phospho-EPIYA-A as shown here. A very few studies have reported generation of phospho-specific α-CagA antibodies designed for one specific EPIYA-motif, although to our knowledge these are not commercially available. A first study showed phosphorylation of EPIYA-motif B after infection and after transfection of CagA from strain NCTC11637 [28]; and another study reported on specific phosphorylation of EPIYA-C in CagA from strains 26695 and P12, including respective phenylalanine substitution controls [22]. In addition, the generation of a phosphospecific antibody against EPIYA-C motif in CagA from strain NCTC11637 was described, but this antibody also recognized the phosphorylated CagA forms of strains GC401 and G501, which lack the EPIYA-motif C, a result suggesting that this antibody may be rather unspecific, able to recognize other phosphorylation sites [30]. Thus, the production of more reliable EPIYA-site specific phospho-antibodies could yield highly valuable research tools.

Our studies focused on the EPIYA-motifs A, B and C of Western *H. pylori* strains. However, it will be also important to investigate the phosphorylation of the generally more potent CagA proteins East-Asian strains with their EPIYA-A, B and D motifs, even though the East-Asian 11-mer EPIYA-D sequence (SPEPIYATIDF) is similar to the Western EPIYA-C sequence (SPEPIYATIDD) [46]. We recently showed that c-Src kinase only phosphorylates CagA EPIYA-C and EPIYA-D motifs, not EPIYA-A and EPIYA-B, using Western blots and the α-PY99 antibody [46]. This result suggests that phospho-EPIYA-D maybe recognized by many or all antibodies that recognize phospho-EPIYA-C. However, this has not yet been tested experimentally, and more studies are certainly warranted to understand the CagA phosphorylation sites in greater detail. A detailed analysis of the various East-Asian EPIYAs is currently underway in our laboratories. One additional option would be to use the phosphopeptide microarray technology to characterize all known individual phospho-EPIYA-motifs and associated amino acid polymorphisms, as was described for human proteins [50], and to test for antibody recognition and host effector protein binding. This would help to better understand the role of single EPIYA-motifs for CagA function and possibly allow correlations and risk predictions for the development of diverse gastric diseases in the future. In addition to CagA, further studies should also focus on the investigation of EPIYA-like phosphorylation sites and downstream signaling used by other bacterial effector proteins from pathogens such as EPEC, *Chlamydia*, *Bartonella, Anaplasma* and *Ehrlichia* species, which collectively represents a fascinating new research area [5], [7]–[13].
